The article "Functions of Heparin Sodium Injection in the Prevention of Peripherally Inserted Central Catheter-Related Venous Thrombosis in NSCLC Patients during Postoperative Chemotherapy" was retracted in 2023. Reasons: signs of a paper mill; suspected computer-generated content; unreliable results or conclusions; concerns about the data.

# Functions of Heparin Sodium Injection in the Prevention of Peripherally Inserted Central Catheter-Related Venous Thrombosis in NSCLC Patients during Postoperative Chemotherapy

**DOI:** 10.1155/2022/1239058

**Published:** 2022-10-17

**Authors:** Shanquan Li, Hong Lu

**Affiliations:** ^1^Venous Catheterization Nursing Clinic, Cancer Hospital Chinese Academy of Medical Sciences, Shenzhen Hospital, Shenzhen, Guangdong Province, China 518100; ^2^Nursing Department, Cancer Hospital Chinese Academy of Medical Sciences, Shenzhen Hospital, Shenzhen, Guangdong Province, China 518100

## Abstract

**Objective:**

This study intended to analyze hazardous factors of venous thrombosis by comparing the effect of different doses of heparin sodium injection on the incidence rate of peripherally inserted central catheter (PICC)-related venous thrombosis in non-small cell lung carcinoma (NSCLC) patients during postoperative chemotherapy.

**Methods:**

425 NSCLC patients who received PICC catheterization in Cancer Hospital Chinese Academy of Medical Sciences, Shenzhen Hospital from July 2019 to July 2021 were collected. Based on their different pathological types, patients were given two different chemotherapy regimens: pemetrexed+cisplatin or paclitaxel+cisplatin. Patients were grouped according to the different doses of heparin sodium injection adopted. Control group (*n* = 140). Catheters were sealed with 10 mL saline only. Group I (*n* = 142). In addition to routine maintenance with normal saline, 2 mL of 10 IU/mL heparin sodium injection was sealed in the catheters under positive pressure every time after catheterization. Group II (*n* = 143). In addition to routine maintenance with normal saline, 5 mL of 10 IU/mL heparin sodium injection was sealed in the same manner as Group I. The baseline characteristics of the three groups of patients were compared by statistical means. Doppler ultrasonography was applied to check the venous thrombosis. The hazardous factors of venous thrombosis were analyzed through correlation analysis and binary logistic regression method.

**Results:**

The incidence rates of thrombosis in the control group, Group I, and Group II were 20.00%, 7.04%, and 2.09%, respectively, with statistically significant differences (*P* < 0.01). Additionally, through the collinear correlation analysis of baseline characteristics, a significant correlation between the dosage of heparin sodium injection and the incidence of thrombosis was observed (*P* < 0.05), but there were no significant differences between other baseline data and the incidence of thrombosis (*P* > 0.05). Binary logistic regression analysis revealed that postoperative use of heparin sodium injection (Group I: OR = 0.312; *P* = 0.003; Group II: OR = 0.082, *P* < 0.001) was a protective factor for preventing thrombosis. In addition, the thromboprophylaxis effect of Group II was better than that of Group I. No serious adverse reactions were found in safety analysis.

The article "Functions of Heparin Sodium Injection in the Prevention of Peripherally Inserted Central Catheter-Related Venous Thrombosis in NSCLC Patients during Postoperative Chemotherapy" was retracted in 2023. Reasons: signs of a paper mill; suspected computer-generated content; unreliable results or conclusions; concerns about the data.

**Conclusion:**

Heparin sodium could significantly lower the incidence rate of PICC-related venous thrombosis in NSCLC patients during postoperative chemotherapy. Heparin sodium injection is safe enough to be promoted among PICC patients with a high risk of venous thrombosis.

## 1. Introduction

Primary bronchial lung cancer is one of the malignancies with high morbidity and mortality in China and the world [1]. With the boosting lung cancer incidence rate, more and more patients are developed with lung cancer, and most of them are diagnosed in the advanced stage with chemotherapy as the main treatment method [2]. Peripherally inserted central catheter (PICC) is a kind of catheterization that send the catheter tip to the bottom third of the superior vena cava, or the junction of the superior vena cava and right atrium, by puncturing the peripheral vein with the catheter. This method allows longer indwelling time, fewer puncture times, and less drug-caused irritation to veins. It provides a long-term effective pathway in veins for the patients who need tumor chemotherapy, long-term intravenous infusion, and inoculation of irritation drugs [3, 4]. Besides, due to easy indwelling and long indwelling time [5, 6], PICC is widely adopted in clinical practice, especially in patients with malignancies who are undergoing chemotherapy [7]. However, what comes next is to prevent catheter-related complications.

PICC-related complications mainly include venous thrombosis, phlebitis, catheter-related bloodstream infection (CRBSI), and catheter ectopy (including abnormal course and abnormal position of blocked catheter tip) [8–12]. Among them, PICC-related venous thromboembolism refers to the process that the blood clots are formed on the inner wall of the vessel where the catheter is located and the adherent wall of the catheter after the placement of PICC, due to factors such as direct damage to the vascular intima by puncturing or catheter and the state of patients themselves. PICC-related venous thrombosis is a common complication of PICC, which is mainly manifested as pain at the involved site, increased body surface temperature, superficial vein exposure, erythema, numbness in the extremities, and impaired neck and limb movements [13]. Multiple publications have exhibited that the incidence of symptomatic PICC-related venous thrombosis is 2%-75% [14, 15], while that of asymptomatic one is as high as 50% [16, 17]. PICC-related venous thrombotic events are also common in patients with lung cancer undergoing chemotherapy. Domestic researchers have reported that the incidence of PICC-related venous thrombosis in lung cancer patients undergoing chemotherapy is 5%-20%, seriously affecting the therapeutic effect [18]. Another work indicated that the incidence of PICC-related venous thrombosis ranged from 3%-30% in lung cancer patients undergoing chemotherapy [19]. Accordingly, preventing the development of PICC-related venous thrombosis and improving the quality of life of patients are urgent. Preventative anticoagulants are clinically applied as a key method to prevent PICC-associated thrombosis in cancer patients [20]. According to research reports, low molecular weight heparin (LMWH), unfractionated heparin (UFH), and warfarin are anticoagulants currently applied in clinical practice, among which, saline-diluted UFH or heparin sodium injection-sealed catheters under positive pressure can effectively prevent microthrombus formation in indwelling catheter [21].

The article "Functions of Heparin Sodium Injection in the Prevention of Peripherally Inserted Central Catheter-Related Venous Thrombosis in NSCLC Patients during Postoperative Chemotherapy" was retracted in 2023. Reasons: signs of a paper mill; suspected computer-generated content; unreliable results or conclusions; concerns about the data.

Effective sealing can effectively prevent blockage, exudation, and catheter-related thrombosis, of which heparin sodium is one of the conventional sealing solutions [22]. Heparin sodium can bind to antithrombin III, enhance the inhibitory effect of antithrombin III on the activation of coagulation factors II, IX, X, XI, and XII, and repress functions of coagulation substances such as thrombin and fibrin, thus exerting anticoagulant effect. Recently, studies have revealed that heparin sodium injection can lower the incidence of venous thrombosis, which is safe and effective. However, a consensus has not been reached on the medication population, medication time, medication dosage, etc.

This study adopted statistical methods to compare the baseline characteristics and the incidence of venous thrombosis of patients treated with different doses of heparin sodium injection. At the same time, the collinearity relationship between the baseline characteristics was analyzed. Then a binary logistic regression analysis was performed to analyze the hazardous factors of thrombosis. In addition, the incidence of adverse reactions of heparin sodium injection was counted, thereby analyzing the safety of the treatment method.

## 2. Data and Methods

### 2.1. General Data

425 NSCLC patients who received PICC catheterization in Cancer Hospital Chinese Academy of Medical Sciences, Shenzhen Hospital from July 2019 to July 2021 were collected. Based on their different pathological types, NSCLC patients were given two different chemotherapy regimens: pemetrexed+cisplatin or paclitaxel+cisplatin. Patients were grouped according to the different heparin sodium injection doses adopted. Control group: 140 patients aged from 28 to 84, including 96 males and 44 females. Their catheters were sealed with only 10 mL saline. Group I: 142 patients aged from 38 to 82, including 114 males and 28 females. In addition to routine maintenance with normal saline, 2 mL of 10 IU/mL heparin sodium injection was sealed in the catheters under positive pressure every time after catheterization. Group II: 143 patients aged from 30 to 84, including 101 males and 42 females. In addition to routine maintenance with normal saline, 5 mL of 10 IU/mL heparin flush injection was sealed in the same manner as Group I. The baseline characteristics of the three groups of patients were compared by statistical methods and were not significantly different (*P* > 0.05) (Table 1). The three groups underwent Doppler ultrasonography on the 7th day after catheterization to check whether venous thrombosis was formed.

The article "Functions of Heparin Sodium Injection in the Prevention of Peripherally Inserted Central Catheter-Related Venous Thrombosis in NSCLC Patients during Postoperative Chemotherapy" was retracted in 2023. Reasons: signs of a paper mill; suspected computer-generated content; unreliable results or conclusions; concerns about the data.

### 2.2. Inclusion Criteria

NSCLC patients who need PICC catheterization for chemotherapy. Their blood biochemistry and coagulation tests should be normal before catheterization. The patient's physique was fair, and The Eastern Cooperative Oncology Group (ECOG) scores were between 0 and 2. All patients had cognitive ability and could respond actively to the treatment. Informed consent was signed.

### 2.3. Exclusion Criteria

Patients with preoperative coagulation disorder, heparin allergy, and active bleeding; patients who took anticoagulant drugs before surgery or had a history of thrombosis; and patients with concomitant heart failure were excluded.

### 2.4. Treatments

Three groups were maintained with normal saline. In the control group, 10 mL normal saline was given each time to seal the catheter 1 to 7 d after catheterization. In Group I, 2 mL of heparin sodium injection (Brand name: Heparin Sodium Injection for Lock Flush, Huabicheng; Specification: 5 mL, 50 units) was sealed in the catheters under positive pressure 1 to 7 d after catheterization. While in Group II, 5 mL of heparin sodium injection was sealed in the same manner as Group I.

### 2.5. Indicators for Observation

All patients included in the study underwent color Doppler ultrasound examination within 6 days, 2w ± 6d, 5w ± 6d, 8w ± 6d since PICC catheterization. Color Doppler ultrasound diagnostic apparatus (German PHILIPS ie3.3, L11-3 probe, 12 MHz) was utilized, to observe whether there were substances attached to the vein that gave out solid mass echo and venous thrombosis at the catheterization site after the catheterization. Thereby the incidence of thrombosis in each group was compared. The incidence of thrombosis refers to the proportion of patients with catheter-related thrombosis in all PICC catheterized patients.

The article "Functions of Heparin Sodium Injection in the Prevention of Peripherally Inserted Central Catheter-Related Venous Thrombosis in NSCLC Patients during Postoperative Chemotherapy" was retracted in 2023. Reasons: signs of a paper mill; suspected computer-generated content; unreliable results or conclusions; concerns about the data.

Thrombosis rate = the number of PICC − related thrombosis within a specified time/the total number of patients with PICC catheterization within the specified time × 100% [23]. It was observed whether there were adverse reactions, hemorrhage or partial bleeding, PICC infections, and other local adverse reactions [24].

### 2.6. Statistical Analysis

SPSS 26.0 software was employed for statistical analysis. Measurement data were analyzed by one-way analysis of variance and examined by LSD-*t* test. Enumeration data underwent chi-square test among groups. *P* < 0.05 (two-sided) implied a statistical significance. The correlation coefficient matrix was obtained by collinearity analysis of the baseline indicators. The relationship between the dosage and venous thrombosis risk was obtained through binary logistic regression.

## 3. Results

### 3.1. Clinical Efficacy

Compared with the control group using normal saline (Table 2), heparin sodium injection significantly reduced the incidence of PICC-related venous thrombosis (*P* < 0.01).

### 3.2. Diagnosis of Collinearity Correlation of Baseline Characteristics

Correlation analysis was performed on patient's group, age, sex, weight, smoking history, ECOG score, pathological type, and operation types (Table 3). The results indicated that different doses of heparin sodium injection were significantly associated with the incidence of venous thrombosis (*P* < 0.05).

### 3.3. Multivariate Binary Logistic Regression

The risk factors or protective factors related to thrombosis were analyzed by multivariate binary logistic regression (Table 4). The results indicated that heparin sodium injection at different doses was a protective factor against thrombosis. Additionally, Group II had the best efficacy (OR = 0.082, 95% CI 0.024-0.277, *P* < 0.001).

### 3.4. Safety

Serious adverse reactions such as deep vein thrombosis (DVT) disease, purpura, skin or systemic allergies, and severe thrombocytopenia were not observed in the three groups of patients.

## 4. Discussion

In recent years, the age of lung cancer patients in China tends to be younger. More than 1.6 million people are diagnosed with lung cancer every year. Venous thromboembolism (VTE) is a common lung cancer complication, mainly including pulmonary embolism (PE) and deep vein thrombosis (DVT) [25]. Connolly et al. [26] indicated that the incidence of VTE in outpatient lung cancer patients reaches 14%. Recent studies have presented that the pathophysiological mechanism of VTE in lung cancer patients is mainly due to the direct activation of coagulation by malignant cells through producing tissue factor (TF), cancer procoagulant (CP), cytokines, and inflammatory factors [27]. By contacting with endothelial cells, platelets, and leukocytes, tumor cells can activate local coagulation, thus promoting platelet activation and aggregation, and stimulating leukocytes to release cytokines [25]. The main risk factors for VTE in patients with lung cancer may be different types and stages of lung cancer, patient factors (history of VTE, elevated platelets, complications (infection, heart failure, etc.)), and tumor treatment measures (radiotherapy, chemotherapy, surgery, and PICC catheterization) [25].

The article "Functions of Heparin Sodium Injection in the Prevention of Peripherally Inserted Central Catheter-Related Venous Thrombosis in NSCLC Patients during Postoperative Chemotherapy" was retracted in 2023. Reasons: signs of a paper mill; suspected computer-generated content; unreliable results or conclusions; concerns about the data.

PICC is commonly used in patients who have malignant tumors and are critically ill because it is beneficial to reduce the risk of drug infiltration, relieving vascular inflammation, avoiding pain caused by repeated punctures, and improving the quality of life of patients. It is suitable for intravenous treatment of home-care patients, thus becoming more popular with medical staff and patients [28, 29]. But recent studies revealed that PICC markedly increased the risks of venous thrombosis [30, 31]. The causes of PICC-related venous thrombosis may be as follows: (1) the diameter of the PICC affects the central flow in the lumen, thereby increasing the risk of turbulent flow and venous thrombosis; (2) the stiffness of the PICC and the direct venous injury and inflammation caused by the insertion, resulting in thrombosis; (3) the introduction of PICC prompts the human body to form a surrounding biofilm to isolate it, coupled with low flow and venous blood stasis, which is conducive to the thrombosis [10]. Hence, both the selection of PICC materials and antithrombotic therapy after surgery are important.

In clinical nursing, heparin is a common drug for effective prevention and treatment of thrombosis [32]. Earlier studies have shown that intravenous heparin is safe and effective for the prevention of recurrent VTE [33]. Heparin is administered by continuous intravenous infusion and subcutaneous injection [34]. Previous randomized trials have shown that there is a correlation between heparin dose and efficacy and safety, although the intensity and duration of anticoagulant effect of heparin is nonlinear with heparin dose [34]. In addition, an increase in heparin dose also increases the risk of bleeding. Therefore, heparin anticoagulation response is commonly monitored clinically by activated partial thromboplastin time (APTT) to adjust continuous intravenous dose [34].

Nevertheless, the clinical dosage of heparin sodium injection is not yet clear. This study confirmed that the 5 mL of 10 IU/mL heparin sodium injection could significantly reduce the incidence of venous thrombosis in NSCLC patients. Additionally, the results of binary logistic regression analysis showed that heparin sodium injection was a protective factor against thrombosis. A study illustrated that old age, obesity, and lung resection are independent predictors of VTE [35]. Through OR analysis, our results showed that age > 63 years (OR = 1.335), weight > 62 kg (OR = 1.303), and smoking history (OR = 1.003) may be risk factors for PICC-related thrombosis, but there was no statistical difference.

The article "Functions of Heparin Sodium Injection in the Prevention of Peripherally Inserted Central Catheter-Related Venous Thrombosis in NSCLC Patients during Postoperative Chemotherapy" was retracted in 2023. Reasons: signs of a paper mill; suspected computer-generated content; unreliable results or conclusions; concerns about the data.

## 5. Conclusion

In summary, the use of heparin sodium injection can improve the coagulation function of patients, facilitate normal blood flow, significantly reduce the occurrence of venous thrombosis, facilitate the surgical treatment of patients, and the survival benefits. This retrospective study still has many shortcomings, including the limited sample size and diversity. In addition, no blood samples were collected for analysis of coagulation parameters and hematology data in our study. Our conclusion calls for further verification by large-sample clinical trials and blood samples in the future.

## Figures and Tables

**Table 1:** Baseline characteristics of patients.

Baseline characteristics	Control group (*n* = 140)	Group I (*n* = 142)	Group II (*n* = 143)	*P* value
Age (years old)	61.88 ± 10.37	61.30 ± 9.10	59.94 ± 10.25	0.243
Sex				0.379
Male	96	114	101	
Female	44	28	42	
Weight (kg)	61.85 ± 7.65	60.63 ± 8.10	60.81 ± 7.68	0.370
Smoking history	70	66	67	0.320
ECOG score	1.06 ± 0.78	1.04 ± 0.78	1.06 ± 0.77	0.973
Pathology type				0.238
Squamous carcinoma	69	68	77	
Adenocarcinoma	71	74	66	
Operation type				0.498
Lung resection	72	72	73	
Lobectomy	68	70	70	

**Table 2:** Comparison of venous thrombosis incidence among groups.

	Control group	Group I	Group II	*P* value
Incidence rates of venous thrombosis	20.00%	7.04%	2.09%	<0.001

**Table 3:** Correlation between incidence of venous thrombosis and baseline characteristics.

Baseline characteristics	Venous thrombosis (*n* = 42)	No venous thrombosis (*n* = 383)	*P* value
Group			**<0.01**
Control group	**28**	**112**	
Group I	**11**	**131**	
Group II	**3**	**140**	
Age			0.373
≤63	20	210	
>63	22	173	
Sex			0.231
Male	34	277	
Female	8	106	
Weight (kg)			0.356
≤62 kg	20		
>62 kg	22	172	
Smoking history			0.528
Yes	22	181	
No	20	202	
ECOG score			0.752
0	10	106	
1	19	151	
2	13	126	
Pathological types			0.354
Squamous carcinoma	24	190	
Adenocarcinoma	18	193	
Operation type			0.613
Lung resection	23	194	
Lobectomy	19	189	

**Table 4:** Results of multivariate binary logistic regression analysis.

Variate	OR	95% CI		*P*
		Lower	Upper	
Group I (group I vs control group)	0.312	0.146	0.665	0.003
Group II (group II vs group II)	0.082	0.024	0.277	<0.001
Group I vs group II	3.824	1.039	14.078	0.044
Age (>63 vs ≤63)	1.335	0.680	2.619	0.401
Sex (female vs male)	0.550	0.234	1.291	0.170
Weight (>62 vs ≤62)	1.303	0.669	2.538	0.436
Smoking history (yes vs no)	1.003	0.505	1.992	0.993
Pathological types (adenocarcinoma vs squamous carcinoma)	0.707	0.356	1.403	0.321
ECOGS = 1 (1 vs 0)	0.739	0.367	1.487	0.396
ECOGS = 2 (2 vs 0)	0.601	0.277	1.302	0.197
Operation type (lobectomy vs lung resection)	0.842	0.428	1.655	0.618

The article "Functions of Heparin Sodium Injection in the Prevention of Peripherally Inserted Central Catheter-Related Venous Thrombosis in NSCLC Patients during Postoperative Chemotherapy" was retracted in 2023. Reasons: signs of a paper mill; suspected computer-generated content; unreliable results or conclusions; concerns about the data.

## Data Availability

The data used to support the findings of this study are included within the article. The data and materials in the current study are available from the corresponding author on reasonable request.
